# The Pharmacological Mechanism of the Effect of Plant Extract Compound Drugs on Cancer Pain Based on Network Pharmacology

**DOI:** 10.1155/2022/9326373

**Published:** 2022-02-27

**Authors:** Yuanyuan Shen, Jun Wang, Pengpeng Yan, Tiantian Chen, Xingrui Li, Ming Jiang

**Affiliations:** Department of Anesthesia, Luoyang Hospital of TCM, Luoyang 471000, China

## Abstract

**Objective:**

We systematically analyzed the mechanism of plant-derived drugs alleviating cancer pain in our hospital through network pharmacology, so as to provide the possibility of further application of traditional Chinese medicine in the treatment of cancer pain.

**Methods:**

We used TCMSP, ETCM, and TCMID databases to mine the active ingredients of plant-derived drugs. We combined OMIM, GeneCards, and DrugBank databases to mine and match the common targets of plant-derived drugs for cancer pain. We used the STRING platform and Cytoscape software to analyze and screen out the core targets. We used GO and KEGG methods to analyze the biological processes, molecular functions, cellular composition, and signaling pathways involved in the reduction of cancer pain by plant-derived drugs.

**Results:**

We found 153 active ingredients from botanical drugs by TCMSP (Traditional Chinese Medicine Systems Pharmacology Database and Analysis Platform, TCMSP), ETCM (The Encyclopedia of Traditional Chinese Medicine), and TCMID (Traditional Chinese Medicine Integrated Database) databases, covering 341 protein targets in human body. Combined with OMIM (Online Mendelian Inheritance in Man), GeneCards, and DrugBank databases, we excavated and matched 141 targets of plant-derived drugs and cancerous pain diseases. Through the analysis of the STRING platform and Cytoscape software, 19 core targets including TNF, MAPK1, JUN, and IL-6 were screened out. Go and KEGG enrichment showed that plant-derived drugs alleviated cancer pain processes involving 193 biological processes, 47 molecular functions, 22 cell components, and 118 signaling pathways. By screening genes involved in KEGG signaling pathway, it was found that plant-derived drugs were mainly associated with PI3K-Akt signaling pathway, tumor necrosis factor signaling pathway, MAPK signaling pathway, Toll-like receptor signaling pathway, and HIF-1 signaling pathway in alleviating cancer pain.

**Conclusion:**

These results indicate that botanical drugs can positively affect the expression of inflammatory factors and apoptotic factors in the process of treatment and relief of cancer pain, which is expected to have a potential therapeutic effect on the relief of cancer pain.

## 1. Introduction

Cancer pain is a chronic pain with a unique and complex mechanism. At the early stage, cancer pain is mainly sensitized by primary afferent nerves caused by a series of pain-causing substances released by tumor cells and inflammatory cells and continuously activated osteoclasts, while at the later stage, cancer pain is mainly caused by nerve compression and injury caused by tumor growth [1]. In recent years, with the aging of the society and the increasing incidence of cancer, about half of the patients with malignant tumors have different degrees of cancer pain, especially the incidence of cancer pain in advanced patients is as high as 60–80%, which seriously affects the patients' disease recovery and quality of life [2]. Cancerous pain is a kind of pain with areas in need of repair or adjustment after the information transmission to the nerve center of feeling, although the clinical use of “three steps” analgesia method can partly control or relieve patients' pain, but as the disease progresses, the tumor load increases, and the increase of the analgesic drug resistance and adverse drug reactions are led to the decrease of the tolerance [3–5].

The understanding of pain in Huangdi Neijing is as follows: “The meridians are not only popular, but also endless around; the cold enters the meridians but delays, and the weeping fails; the blood is little outside the veins, and the qi is blocked in the middle, so the death is painful.” Chinese medicine research believes that cancer pain is cancer toxin cohesion, meridian block blockage, and not general pain. If the human body is in a state of qi deficiency, it can not nourish the viscera and meridians, so pain will occur. Pain and its treatment are the diseases that are first felt and recognized by human beings. In other words, after the body is stimulated by the internal and external environment, pain-causing substances are generated and released from the tissues, pain receptors are sensitized, pain information is transmitted, sensory center perceives, and finally, pain enters the consciousness stage, which leads to pain [6]. Among them, pain-causing substances include bradykinin, histamine, 5-HT, and prostaglandin, which can excite or sensitize the receptors when they are stimulated by various stimuli [7]. At present, western medicine is widely used in the treatment of various kinds of pain, which has the effect of addiction and tolerance, which limits the clinical application and reduces the therapeutic effect [8, 9]. The application of traditional Chinese medicine in the treatment of pain has a history of thousands of years. In ancient books and modern scientific research, it has been proved that more than 800 kinds of traditional Chinese medicine can effectively relieve pain [10, 11]. Traditional Chinese medicine compound has the characteristics of multiherbs, multicomponents, and multitarget coordination, but the current research methods cannot fully explain its effects. Network pharmacology, from a macroscopic and systematic perspective, explores the overall effect of drug treatment on diseases, breaking the previous research mode of single compound and single target, and providing a new idea for the study of the TCM compound. There are 11 herbal medicines of plant origin, including Astragalus membranaceus, Poria cocos, honeysuckle, Cyperus, Paeonia lactiflora, bupleurum, Hedyotis diffusa, Scutellaria barbata, Trichosanthes kirilowii, Arisaema, and Scutellaria baicalensis. Among them, Astragalus membranaceus, Poria cocos, Cyperus, Paeonia lactiflora, and Scutellaria baicalensis have been used many times in the clinical research of pain treatment . However, the specific mechanism of pain relief by botanical drugs is still unclear. In order to optimize the clinical therapeutic effect of botanical drugs and clarify its mechanism of action, we obtained the effective chemical components and corresponding targets through TCMSP, ETCM, TCMID, and other databases; screened the pain-related targets from GeneCards, OMIM, DrugBank, and other databases; and constructed the “humanized” model by using Cytoscape software and STRING database. To screen the key components and key targets of therapeutic effect, GO and KEGG pathway enrichment analysis was carried out on the key targets through the DAVID platform, and the potential mechanism of 11 herbal extracts was obtained [12–18].

## 2. Materials and Methods

### 2.1. Identification and ADME Screening of Candidate Compounds of Traditional Chinese Medicine

In this study, all the active ingredients of 11 herbal medicines of botanical origin were searched by TCMSP, ETCM, and TCMID [19, 20]. The names of 11 traditional Chinese medicines, Astragalus membranaceus, Poria cocos, Honeysuicerae lonicerae, Radix Paeoniae lactiflora, Radix Bupleurum, Hedyotis diffusa, Scutellaria scleroides, Fructus Trichosanthis, Araceae aratidae, Radix Scutellariae, were input, and the main active components were further screened according to the oral availability (OB) ≥30% and drug-like properties (DL) ≥0.18. OB and DL are the key indicators to evaluate the effective availability of drugs. Generally speaking, active ingredients with OB ≥ 30% and DL ≥ 0.18 can be regarded as the main active ingredients of drugs [21].

### 2.2. Prediction of Related Targets of Active Compounds in Traditional Chinese Medicine

TCMSP, PharmMapper, SwissTarget, and other databases were used to screen the protein targets corresponding to the main active components of the abovementioned traditional Chinese medicine [22]. By using the retrieval function of UniproKBT in the UniProt database [23], all target gene names were corrected into official gene symbol names by inputting protein names, and active ingredients without targets were removed to obtain the information of active ingredients and related targets.

### 2.3. Cancer Pain Disease Targets and Protein Collection

According to DrugBank, GeneCards, and OMIM databases, the English “cancer pain” corresponding to pain was used as the key word to search and screen the related targets, and the targets of three disease databases were combined to remove the repetitive base, so as to obtain the potential targets of pain, and by using the retrieval function of UniProKBT in the UniProt database and by inputting the name of protein and limiting the species to human, all the potential targets of pain were identified. The name of target gene was corrected to official gene symbol, and the active components without target were eliminated to obtain the final disease target [24, 25].

### 2.4. Construction of “Compound-Target-Cancerous Pain” Signaling Pathway

The protein-protein interaction (PPI) network of potential targets and disease targets was constructed by using Cytoscape 3.7.2, and the two network graphs were fused and the intersection network was extracted by using the correlation function in the software. The direct and indirect target regulatory networks of 14 herbal medicines for cancer pain relief were obtained.

### 2.5. GO and KEGG Analysis

In order to clarify the potential action targets of active ingredients in 14 herbal medicines of plant origin, as well as the role of cancer-related pain targets in gene function and signaling pathway, GO and KEGG enrichment analysis was conducted in the DAVID database and Metascape platform based on annotation and visualization modules [26]. In this study, *R* language programming was used for GO and KEGG pathway analysis, and set thresholds *P* < 0.05. The possible mechanism of analgesic effects of 14 herbal herbs derived from plants was predicted through gene enrichment analysis, and the results were imported into the mapping software for visual mapping [27] (Table 1).

## 3. Results

### 3.1. Analysis of Components and ADME of Botanical Drugs

By searching TCMSP, ETCM, and TCMID databases and analyzing ADME, based on OB ≥ 30% and DL ≥ 0.18, a total of 154 active components were obtained from 11 kinds of herbal medicines, including 23 Astragalus membranaceus, 20 Poria cocos, 26 Honeysuckle, 18 Cyperus, 13 Paeonia alba, 17 Bupleurum, 7 Hedyotis diffusa, 29 Scutellaria barbata, 11 Trichosanthes kirilowii, 7 Arisaema, and 36 Scutellaria baicalensis. The compound information of 11 Traditional Chinese medicines is shown in Figure 1 and Table 2–12 [28].

### 3.2. Target Prediction of Active Components in Traditional Chinese Medicine

Through TCMSP, PharmMapper, SwissTarget database retrieval, and comparison with the UniProt database, a total of 341 protein targets of 153 active components of botanical drugs were obtained, including 247 Astragalus, 94 Poria cocos, 262 Honeysuckle, 178 Cyperus, 72 Paeonia lactiflora, 148 Hupleurum, 153 Hedyotis diffusa, 178 Scutellaria barbata, 9 Trichosanthes kirilowii, 39 Arisaema, and 90 Scutellaria baicalensis. The protein target information of 11 active components of traditional Chinese medicine is shown in Figure 2.

### 3.3. Screening of Pain-Related Targets

Based on OMIM, GeneCards, and DrugBank databases, pain disease-related targets were screened with “cancer pain” as the key word. The results showed that there were 670 pain disease-related targets in the OMIM database, 1086 GeneCards database, and 215 DrugBank database. A total of 1695 targets were obtained from the three databases. Compared with the UniProt database, 1110 verified human pain disease-related targets were obtained. By matching 341 protein targets of active components of plant-derived drugs, 141 common targets of plant-derived drugs and cancer pain diseases were obtained. The Venn diagram and detailed target information are shown in Figure 3 and Table 13, respectively.

### 3.4. PPI Network Construction

The interaction network of 141 potential targets was constructed by using the STRING database platform. The minimum interaction threshold was set to “0.9,” and the results are shown in Figure 4. The nodes in the figure are intersection genes, and the edges represent the association degree of the intersection genes, and the thickness represents the binding degree. As shown in the figure, there are 140 nodes and 538 edges. The PPI network diagram is imported into the software Cytoscape 3.7.2, and the network pictures are analyzed by tools. We selected those targets with greater than average degree and betweenness centrality, a total of 19 targets, as potential key targets for plant-derived drugs to exert analgesic effects The main proteins closely related to analgesic effect of botanical drugs are TNF, mapk1, Jun, and IL-6, as shown in Figure 5 and Table 14.

### 3.5. Construction of “Compound Traditional Chinese Medicine Compound Target Disease” Network Diagram of Analgesic Effect of Botanical Drugs

Nineteen core targets of botanical drug analgesia were obtained from 2.4, and the corresponding compounds and traditional Chinese medicine were screened and matched. The network diagram of “compound traditional Chinese medicine compound target disease” of botanical drug analgesia was predicted by using Cytoscape 3.7.2 software. The results are shown in Figures 6 and 7.

### 3.6. GO and KEGG Enrichment Analysis

Through DAVID and STRING databases, 141 targets of botanical drug pain disease were enriched and analyzed, including biological process (BP), molecular function (MF), and cell composition (CC). There are 193 biological processes, 47 molecular functions, and 22 cell components; 20 enriched genes are selected and mapped through the mapping software, as shown in Figure 8; 118 signaling pathways are involved in KEGG pathway abdominal muscle analysis, and 20 enriched genes are screened according to the number of enriched genes, as shown in Figure 9.

## 4. Discussion

Modern medicine believes that cancer pain is mainly caused by the disease itself or the pain caused in the treatment process. Tumors infiltrate bone tissue, and bone tissue destruction results in the release of prostaglandins. It invades the viscera, causing vasospasm, occlusion, and eventually necrosis of the viscera. Or it may compress peripheral nerves, nerve roots, spinal cord, etc. The patient's own mental tension and psychological pressure can cause pain disorders. There is no name for cancer pain in Chinese medicine, but according to the pain of different parts of cancer, it can be assigned to the pain syndrome of the corresponding parts. For example, pain caused by brain tumor, nasopharyngeal cancer, and cancer brain metastasis is classified as “headache.” Cancer of the esophagus and lung can be classified as “chest pain.” Pain caused by gastric cancer is classified as “stomachache.” Pain caused by liver cancer is classified as “flank pain.” Pain caused by pancreatic and colorectal cancer is classified as “abdominal pain.” The pain caused by bone cancer and cancer bone metastasis is classified as “Bi syndrome” or “Gubi syndrome.”

Pain is a kind of feeling of human disease caused by tissue injury, which stimulates the sensory system [29]. It is of great significance and research value in clinical diagnosis and treatment. Usually, the clinical pain mainly comes from the noxious stimulation of internal and external conditions caused by disease or surgery, which not only includes the defense response of the human body to noxious stimulation, but also a clinical manifestation of a variety of diseases and postoperative reactions [30]. Most of the patients have severe pain or chronic long-term pain and need to be treated with analgesic drugs. Cancer pain usually accompanies the whole course of cancer patients, so that patients are in pain, anxiety and even depression, and other negative emotions for a long time, causing some patients to lose confidence in life, which seriously affects the quality of life of patients. Therefore, how to effectively control the degree of cancer pain of cancer patients has great significance for the treatment of cancer and the improvement of life quality of cancer patients [31, 32]. We need to understand the meaning of this. Therefore, the research of analgesic drugs has become one of the hot directions of modern drug research, but the clinical use of chemical drugs for acute or chronic pain, such as opioids and nonopioids: morphine, codeine, pethidine, aspirin, indomethacin, ibuprofen, and so on [33]. Although the above methods have achieved good clinical efficacy, the side effects are often more serious due to the continuous and large dose of use. Traditional Chinese medicine believes that pain is due to body deficiency, deficiency of healthy qi, and invasion of external pathogens, which eventually leads to heat toxin and internal stagnation, obstruction of meridians and collaterals, qi stagnation, and blood stasis. Herbal medicine is one of the most important methods of traditional Chinese medicine in treating cancer pain, and studies have shown that bitter cold herbal medicine has exact antitumor effect, with less toxic and side effects and obvious effect [34, 35]. The clinical analgesic effect of chemical drugs has been fully recognized, but for patients with chronic pain, long-term use will produce dependence, peptic ulcer, and other adverse reactions. Accordingly, with the development of traditional Chinese medicine industry, the research of natural plant extracts for pain treatment is gradually deepening [36, 37].

Botanical medicine is an important method for the treatment of cancer pain. This method should be highly valued by medical staff. External application of traditional Chinese medicine is directly administered to patients on the body surface of medical staff. Under the condition of absorption on the skin or mucous membrane surface of the patient, it can reach the pain site of the patient, produce good analgesic effect, and gradually reduce the side effects caused by oral drugs [38]. In this study, 11 plant-derived drugs widely used in clinical pain treatment were selected as follows: Astragalus membranaceus, Poria cocos, Honeysuckle, Cyperus, Paeonia lactiflora, Bupleurum, Hedyotis diffusa, Scutellaria barbata, Trichosanthes kirilowii, Arisaema, and Scutellaria baicalensis. Among them, Astragalus is sweet in taste and mild in nature. It is mainly used for blood numbness of limbs and hemiplegia. Poria cocos is sweet and light, and has a mild nature. Honeysuckle has the characteristics of sweet-cold clearing, light aroma, and drooping, is good for clearing away heat and detoxification, and treats carbuncle sores and boils. Cyperus is pungent, relieves bitterness, and tastes sweet, and it is harmonious, smooth, and unbiased, and works well for soothing the liver, regulating qi, and relieving pain. Paeonia lactiflora has sour, sweet, and bitter taste, it is mild cold in nature, and it has the effect of softening the liver and relieving pain. Bupleurum is bitter and mildly cold, and aromatic, relieves diarrhea, and mainly treats flank pain, irregular menstruation, and dysmenorrhea. Hedyotis diffusa is bitter and cold to clear diarrhea, and sweet and cold to infiltrate and benefit, clear away heat and toxins, dissipate carbuncle, treat sore carbuncle, sore throat, and intestinal carbuncle. Scutellaria barbata has a pungent flavor that can disperse, relieve bitter cold, and clear diarrhea, not only dissipate blood stasis and cool blood to stop bleeding, but also clear heat and water to relieve drenching and swelling, and it is good at treating sores and cancers. Trichosanthes kirilowii is sweet and cold lubricating, and has the effect of clearing lungs, moisturizing dryness and resolving phlegm, reducing swelling, and relieving lumps. Arisaema has bitterness, dryness, and strong medicinal power, and it is especially good at dispelling meridian wind and phlegm, not only drying dampness and reducing phlegm, but also dispelling wind and relieving spasm. Scutellaria baicalensis is bitter cold, clears venting and dryness, and can cool blood and stop bleeding [39, 40].

Based on the database of TCMSP, ETCM and TCMID, and OB ≥ 30% and DL ≥ 0.18, 23 Astragalus membranaceus, 20 Poria cocos, 26 Honeysuckle, 18 Cyperus, 13 Paeonia lactiflora, 17 Bupleurum, 7 Hedyotis diffusa, 29 Scutellaria barbata, 11 Trichosanthes kirilowii, 7 Arisaema, and 36 Scutellaria baicalensis were obtained, with a total of 154 active components. Through TCMSP, PharmMapper, SwissTarget database retrieval, and comparison with the UniProt database, 341 protein targets of plant-derived drugs were obtained. Through 1110 targets related to human pain diseases, 141 common targets of plant-derived drugs pain diseases were obtained. The interaction network of 141 potential targets was constructed by using the STRING database platform, and the PPI network diagram was imported into Cytoscape 3.7.2 in the software, the network images were analyzed by tools, and the 19 targets with degree and betweenness centrality >15 were the potential key targets for the analgesic effect of botanical drugs. The main proteins closely related to the analgesic effect of botanical drugs were TNF, MAPK1, JUN, IL-6, and so on. GO enrichment analysis by the DAVID platform showed that the mechanism of pain relief by botanical drugs mainly involved 193 biological processes, 47 molecular functions, and 22 cell components; 118 signaling pathways were obtained by the abdominal muscle analysis of the KEGG pathway. The main biological processes are as follows: RNA polymerase II promoter, transcriptional DNA template, inflammatory reaction, transcriptional positive regulatory DNA template, apoptosis process, immune reaction, active regulation of angiogenesis, regulation of cell proliferation, activation of cysteine-type endopeptidase activity, regulation of apoptosis process, steroid hormone-mediated signaling pathway, lipopolysaccharide-mediated signaling pathway, and sequence-specific DNA binding transcription, positive regulation of NF-kappa B transcription factor activity, negative regulation of cell proliferation, negative regulation of transcription, and so on. Cell components include nucleus, cytoplasm, extracellular space, extracellular exosomes, cytosol, organic components of plasma membrane, intracellular mitochondria, external plasma membrane, endoplasmic reticulum, cell surface, extracellular matrix, postsynaptic membrane, complex receptors, membrane rafts, neuronal projection, cell junction, nuclear chromatin, spindle, RNA polymerase II transcription factor complexThings. Molecular functions include zinc ion binding, ATP binding transcription factor activity, DNA binding, heme node, cytokine activity, protein dimer activity, RNA polymerase II core promoter proximal region-specific sequence DNA binding, chromatin binding, steroid hormone receptor activity, growth factor activity, iron ion binding, transcriptional activator activity, steroid binding, transcriptional regulatory region DNA binding, amino acid endopeptidase activity, adrenaline binding, monooxygenase activity metalloendopeptidase activity, norepinephrine binding, aromatase activity, tumor necrosis factor receptor binding, MAPK activity, peroxidase activity, transmembrane receptor protein tyrosine kinase activity, core promoter sequence-specific DNA binding, drug binding, and chemokine activity. KEGG signaling pathways mainly include cancer, hepatitis B, PI3K-Akt signaling pathway, proteoglycan in cancer, influenza, tumor necrosis factor signaling pathway, pulmonary tuberculosis, MAPK signaling pathway, HTLV-I, toxoplasmosis infection, prostate cancer, Toll-like receptor signaling pathway, adhesive plaque, HIF-1 signaling pathway, hepatitis C, Ras signaling pathway, pancreatic cancer, small cell lung cancer, T-cell receptor signaling pathway, osteoclast differentiation, nonalcoholic fatty liver disease (NAFLD), herpes simplex infection, and cAMP signaling pathway ssc05206: microRNAs in tumors. It can be seen from the above signaling pathways that plant-derived drugs not only regulate the expression of inflammatory factors through inflammatory signaling pathways to relieve pain, but also actively participate in prostate cancer, pancreatic cancer, small cell lung cancer, and other cancer pathways, in order to achieve the effect of relieving cancer pain.

## 5. Conclusion

In conclusion, the material basis and the possible mechanism of action of the active components of plant-derived drugs were preliminarily discussed through network pharmacology. In this article, the effective chemical components and corresponding targets of plant-derived drugs were obtained by TCMSP, ETCM, TCMID, and other databases. GeneCards, OMIM, DrugBank, and other databases were used to screen out pain-related targets. Cytoscape software and STRING database were used to construct the “compound target” interaction network and protein interaction (PPI) network to screen the key components and key targets for therapeutic effects. GO and KEGG pathway enrichment analysis was performed on key targets through the DAVID platform, and the potential action mechanism of 11 herbal extracts of plant origin drugs was learned. We found 153 active ingredients from botanical drugs by TCMSP, ETCM, and TCMID databases, covering 341 protein targets in the human body. Combined with OMIM, GeneCards, and DrugBank databases, we excavated and matched 141 targets of plant-derived drugs and cancerous pain diseases. Through the analysis of the STRING platform and Cytoscape software, 19 core targets including TNF, MAPK1, JUN, and IL-6 were screened out. Go and KEGG enrichment showed that plant-derived drugs alleviated cancer pain processes involving 193 biological processes, 47 molecular functions, 22 cell components, and 118 signaling pathways. By screening genes involved in the KEGG signaling pathway, it was found that plant-derived drugs were mainly associated with PI3K-Akt signaling pathway, tumor necrosis factor signaling pathway, MAPK signaling pathway, Toll-like receptor signaling pathway, and HIF-1 signaling pathway in alleviating cancer pain. These results indicate that botanical drugs can positively affect the expression of inflammatory factors and apoptotic factors in the process of treatment and relief of cancer pain, which is expected to have a potential therapeutic effect on the relief of cancer pain. Although TCMSP and other databases were used to obtain the chemical components of plant-derived drugs, these data are not complete. In the later stage, UPLC, UPLC-Q-TOF-MS, and other methods should be used to detect the chemical components of plant-derived drugs, in order to obtain more comprehensive chemical information to study the mechanism of action of traditional Chinese medicine monomer.

## Figures and Tables

**Figure 1:** Network of botanical drugs, traditional Chinese medicine, and compounds.

**Figure 2:** Network of traditional Chinese medicine active ingredients target.

**Figure 3:** Venn map of target. ((a) is the Venn map of cancer pain-related targets in OMIM, GeneCards, and DrugBank databases; (b) is the Venn map of common targets of botanical drugs and cancer pain diseases).

**Figure 4:** PPI network of botanical drugs cancer pain diseases.

**Figure 5:** Core target map of different parameters of botanical drug cancer pain disease (selectivity and betweenness centrality are (a) 30; (b) 25; (c) 20; (d) 15).

**Figure 6:** Traditional Chinese medicine target disease network.

**Figure 7:** Compound Chinese medicine compound target disease network.

**Figure 8:** Enrichment analysis of GO in pain target of botanical drugs.

**Figure 9:** Enrichment analysis of the KEGG pathway, a pain target of botanical drugs.

**Table 1:** Website of database and network platform.

TCMSP	https://tcmspw.com/tcmsp.php
ETCM	http://www.tcmip.cn/ETCM/index.php/
TCMID	http://www.Megabionet.org/tcmid/
PharmMapper	http://lilab-ecust.cn/pharmmapper/
SwissTarget	http://new.swisstargetprediction.ch/
UniProt	https://www.uniprot.org/
DrugBank	https://omim.org/
GeneCards	https://omim.org/
OMIM	https://omim.org/
DAVID	https://metascape.org/gp/
Metascape	https://metascape.org/gp/
STRING	https://string-db.org/

**Table 2:** Related information of active components of Astragalus membranaceus.

Mol ID	Molecule name	OB (%)	DL

MOL000211	Mairin	55.38	0.78
MOL000239	Jaranol	50.83	0.29
MOL000296	Hederagenin	36.91	0.75
MOL000033	24-Propylcholesterol	36.23	0.78
MOL000354	Isorhamnetin	49.60	0.31
MOL000371	3,9-Di-O-methylnissolin	53.74	0.48
MOL000374	5′-Hydroxyiso-muronulatol-2′,5′-di-O-glucoside	41.72	0.69
MOL000378	7-O-Methylisomucronulatol	74.69	0.30
MOL000379	9,10-Dimethoxypterocarpan-3-O-*β*-D-glucoside	36.74	0.92
MOL000380	(6aR,11aR)-9,10-Dimethoxy-6a,11a-dihydro-6H-benzofurano[ [2, 3]-c]chromen-3-ol	64.26	0.42
MOL000387	Bifendate	31.10	0.67
MOL000392	Formononetin	69.67	0.21
MOL000398	Isoflavanone	109.99	0.30
MOL000417	Calycosin	47.75	0.24
MOL000433	FA	68.96	0.71
MOL000438	(3R)-3-(2-Hydroxy-3,4-dimethoxyphenyl)chroman-7-ol	67.67	0.26
MOL000439	Isomucronulatol-7,2′-di-O-glucosiole	49.28	0.62
MOL000442	1,7-Dihydroxy-3,9-dimethoxy pterocarpene	39.05	0.48
MOL000098	Quercetin	46.43	0.28
MOL000359	Sitosterol	36.91	0.75
MOL000433	Folic acid	68.96	0.71
MOL000239	Kumatakenin	50.83	0.29
MOL002565	Medicarpin	49.22	0.34

**Table 3:** Related information of active components of Poria cocos.

Mol ID	Molecule name	OB (%)	DL

MOL000273	(2R)-2-[(3S,5R,10S,13R,14R,16R,17R)-3,16-Dihydroxy-4,4,10,13,14-pentamethyl-2,3,5,6,12,15,16,17-octahydro-1H-cyclopenta[a]phenanthren-17-yl]-6-methylhept-5-enoic acid	30.93	0.81
MOL000275	Trametenolic acid	38.71	0.80
MOL000276	7,9(11)-Dehydropachymic acid	35.11	0.81
MOL000279	Cerevisterol	37.96	0.77
MOL000280	Dehydrotumulosic acid	31.07	0.82
MOL000282	Ergosta-7,22E-dien-3beta-ol	43.51	0.72
MOL000283	Ergosterol peroxide	40.36	0.81
MOL000285	Polyporenic acid C	38.26	0.82
MOL000287	3*β*-Hydroxy-24-methylene-8-lanostene-21-oic acid	38.70	0.81
MOL000289	Pachymic acid	33.63	0.81
MOL000290	Poricoic acid A	30.61	0.76
MOL000291	Poricoic acid B	30.52	0.75
MOL000292	Poricoic acid C	38.15	0.75
MOL000296	Hederagenin	36.91	0.75
MOL000300	Dehydroeburicoic acid	44.17	0.83
MOL000289	Pachymic acid	33.63	0.81
MOL000290	Poricoic acid A	30.61	0.76
MOL000291	Poricoic acid B	30.52	0.75
MOL000292	Poricoic acid C	38.15	0.75
MOL000275	Trametenolic acid	38.71	0.80

**Table 4:** Related information of active components of honeysuckle.

Mol ID	Molecule name	OB (%)	DL

MOL001494	Mandenol	42.00	0.19
MOL001495	Ethyl linolenate	46.10	0.20
MOL002707	Phytofluene	43.18	0.50
MOL002914	Eriodyctiol (flavanone)	41.35	0.24
MOL003006	(-)-(3R,8S,9R,9aS,10aS)-9-Ethenyl-8-(beta-D-glucopyranosyloxy)-2,3,9,9a,10,10a-hexahydro-5-oxo-5H,8H-pyrano[ [3, 4]-d]oxazolo[ [2, 3]-a]pyridine-3-carboxylic acid_qt	87.47	0.23
MOL003014	Secologanic dibutylacetal_qt	53.65	0.29
MOL002773	Beta-carotene	37.18	0.58
MOL003036	ZINC03978781	43.83	0.76
MOL003044	Chryseriol	35.85	0.27
MOL003059	Kryptoxanthin	47.25	0.57
MOL003062	4,5′-Retro-.beta.,.beta.-Carotene-3,3′-dione, 4′,5′-didehydro-	31.22	0.55
MOL003095	5-Hydroxy-7-methoxy-2-(3,4,5-trimethoxyphenyl)chromone	51.96	0.41
MOL003101	7-Epi-Vogeloside	46.13	0.58
MOL003108	Caeruloside C	55.64	0.73
MOL003111	Centauroside_qt	55.79	0.50
MOL003117	Ioniceracetalides B_qt	61.19	0.19
MOL003124	Xylostosidine	43.17	0.64
MOL003128	Dinethylsecologanoside	48.46	0.48
MOL000358	Beta-sitosterol	36.91	0.75
MOL000422	Kaempferol	41.88	0.24
MOL000449	Stigmasterol	43.83	0.76
MOL000006	Luteolin	36.16	0.25
MOL000098	Quercetin	46.43	0.28
MOL000359	Sitosterol	36.91	0.75
MOL000296	Hederagenin	36.91	0.75
MOL003044	Chrysoeriol	35.85	0.27

**Table 5:** Related information of active components of cyperus.

Mol ID	Molecule name	OB (%)	DL

MOL003044	Chryseriol	35.85	0.27
MOL000354	Isorhamnetin	49.60	0.31
MOL003542	8-Isopentenyl-kaempferol	38.04	0.39
MOL000358	Beta-sitosterol	36.91	0.75
MOL000359	Sitosterol	36.91	0.75
MOL004027	1,4-Epoxy-16-hydroxyheneicos-1,3,12,14,18-pentaene	45.10	0.24
MOL004053	Isodalbergin	35.45	0.20
MOL004058	Khell	33.19	0.19
MOL004059	Khellol glucoside	74.96	0.72
MOL010489	Resivit	30.84	0.27
MOL004068	Rosenonolactone	79.84	0.37
MOL004071	Hyndarin	73.94	0.64
MOL004074	Stigmasterol glucoside_qt	43.83	0.76
MOL004077	Sugeonyl acetate	45.08	0.20
MOL000422	Kaempferol	41.88	0.24
MOL000449	Stigmasterol	43.83	0.76
MOL000006	Luteolin	36.16	0.25
MOL000098	Quercetin	46.43	0.28

**Table 6:** Related information of active components of *Paeonia lactiflora*.

Mol ID	Molecule name	OB (%)	DL

MOL001910	11-Alpha,12-alpha-epoxy-3beta-23-dihydroxy-30-norolean-20-en-28,12beta-olide	64.77	0.38
MOL001918	Paeoniflorgenone	87.59	0.37
MOL001919	(3S,5R,8R,9R,10S,14S)-3,17-Dihydroxy-4,4,8,10,14-pentamethyl-2,3,5,6,7,9-hexahydro-1H-cyclopenta[a]phenanthrene-15,16-dione	43.56	0.53
MOL001921	Lactiflorin	49.12	0.80
MOL001924	Paeoniflorin	53.87	0.79
MOL001925	paeoniflorin_qt	68.18	0.40
MOL001928	albiflorin_qt	66.64	0.33
MOL001930	Benzoyl paeoniflorin	31.27	0.75
MOL000211	Mairin	55.38	0.78
MOL000358	Beta-sitosterol	36.91	0.75
MOL000359	Sitosterol	36.91	0.75
MOL000422	Kaempferol	41.88	0.24
MOL000492	(+)-Catechin	54.83	0.24

**Table 7:** Related information of active components of bupleurum.

Mol ID	Molecule name	OB (%)	DL

MOL001645	Linoleyl acetate	42.10	0.20
MOL002776	Baicalin	40.12	0.75
MOL000449	Stigmasterol	43.83	0.76
MOL000354	Isorhamnetin	49.60	0.31
MOL000422	Kaempferol	41.88	0.24
MOL004598	3,5,6,7-Tetramethoxy-2-(3,4,5-trimethoxyphenyl)chromone	31.97	0.59
MOL004609	Areapillin	48.96	0.41
MOL013187	Cubebin	57.13	0.64
MOL004624	Longikaurin A	47.72	0.53
MOL004628	Octalupine	47.82	0.28
MOL004644	Sainfuran	79.91	0.23
MOL004648	Troxerutin	31.60	0.28
MOL004653	(+)-Anomalin	46.06	0.66
MOL004702	Saikosaponin c_qt	30.50	0.63
MOL004718	*α*-Spinasterol	42.98	0.76
MOL000490	Petunidin	30.05	0.31
MOL000098	Quercetin	46.43	0.28

**Table 8:** Related information of active components of *Hedyotis diffusa*.

Mol ID	Molecule name	OB (%)	DL

MOL001646	2,3-Dimethoxy-6-methyanthraquinone	34.86	0.26
MOL001659	Poriferasterol	43.83	0.76
MOL001663	Oleanolic acid	32.03	0.76
MOL001670	2-Methoxy-3-methyl-9,10-anthraquinone	37.83	0.21
MOL000449	Stigmasterol	43.83	0.76
MOL000358	Beta-sitosterol	36.91	0.75
MOL000098	Quercetin	46.43	0.28

**Table 9:** Related information of active components of Scutellaria barbata.

Mol ID	Molecule name	OB (%)	DL

MOL001040	(2R)-5,7-Dihydroxy-2-(4-hydroxyphenyl)chroman-4-one	42.36	0.21
MOL012245	5,7,4′-Trihydroxy-6-methoxyflavanone	36.63	0.27
MOL012246	5,7,4′-Trihydroxy-8-methoxyflavanone	74.24	0.26
MOL012248	5-Hydroxy-7,8-dimethoxy-2-(4-methoxyphenyl)chromone	65.82	0.33
MOL012250	7-Hydroxy-5,8-dimethoxy-2-phenyl-chromone	43.72	0.25
MOL012251	Chrysin-5-methylether	37.27	0.20
MOL012252	9,19-Cyclolanost-24-en-3-ol	38.69	0.78
MOL002776	Baicalin	40.12	0.75
MOL012254	Campesterol	37.58	0.71
MOL000953	CLR	37.87	0.68
MOL000358	Beta-sitosterol	36.91	0.75
MOL012266	Rivularin	37.94	0.37
MOL001973	Sitosteryl acetate	40.39	0.85
MOL012269	Stigmasta-5,22-dien-3-ol-acetate	46.44	0.86
MOL012270	Stigmastan-3,5,22-triene	45.03	0.71
MOL000449	Stigmasterol	43.83	0.76
MOL000173	Wogonin	30.68	0.23
MOL001735	Dinatin	30.97	0.27
MOL001755	24-Ethylcholest-4-en-3-one	36.08	0.76
MOL002714	Baicalein	33.52	0.21
MOL002719	6-Hydroxynaringenin	33.23	0.24
MOL002915	Salvigenin	49.07	0.33
MOL000351	Rhamnazin	47.14	0.34
MOL000359	Sitosterol	36.91	0.75
MOL005190	Eriodictyol	71.79	0.24
MOL005869	Daucostero_qt	36.91	0.75
MOL000006	Luteolin	36.16	0.25
MOL008206	Moslosooflavone	44.09	0.25
MOL000098	Quercetin	46.43	0.28

**Table 10:** Related information of active components of Trichosanthes kirilowii.

Mol ID	Molecule name	OB (%)	DL

MOL001494	Mandenol	42.00	0.19
MOL002881	Diosmetin	31.14	0.27
MOL004355	Spinasterol	42.98	0.76
MOL005530	Hydroxygenkwanin	36.47	0.27
MOL006756	Schottenol	37.42	0.75
MOL007165	10*α*-Cucurbita-5,24-diene-3*β*-ol	44.02	0.74
MOL007171	5-Dehydrokarounidiol	30.23	0.77
MOL007172	7-Oxo-dihydrokaro-unidiol	36.85	0.75
MOL007175	Karounidiol 3-o-benzoate	43.99	0.50
MOL007179	Linolenic acid ethyl ester	46.10	0.20
MOL007180	Vitamin-e	32.29	0.70
MOL013146	8,11,14-Docosatrienoic acid, methyl ester	43.23	0.30
MOL013156	[(2R)-2-[[[(2R)-2-(Benzoylamino)-3-phenylpropanoyl]amino]methyl]-3-phenylpropyl] acetate	38.88	0.56
MOL001510	24-Epicampesterol	37.58	0.71
MOL000358	Beta-sitosterol	36.91	0.75
MOL000359	Sitosterol	36.91	0.75
MOL000449	Stigmasterol	43.83	0.76
MOL000953	CLR	37.87	0.68

**Table 11:** Related information of active components of Rhizoma Arisaema.

Mol ID	Molecule name	OB (%)	DL

MOL013146	8,11,14-Docosatrienoic acid, methyl ester	43.23	0.30
MOL013156	[(2R)-2-[[[(2R)-2-(Benzoylamino)-3-phenylpropanoyl]amino]methyl]-3-phenylpropyl] acetate	38.88	0.56
MOL001510	24-Epicampesterol	37.58	0.71
MOL000358	Beta-sitosterol	36.91	0.75
MOL000359	Sitosterol	36.91	0.75
MOL000449	Stigmasterol	43.83	0.76
MOL000953	CLR	37.87	0.68

**Table 12:** Related information of active components of *Scutellaria baicalensis* Georgi.

Mol ID	Molecule name	OB (%)	DL

MOL001689	Acacetin	34.97	0.24
MOL000173	Wogonin	30.68	0.23
MOL000228	(2R)-7-Hydroxy-5-methoxy-2-phenylchroman-4-one	55.23	0.20
MOL002714	Baicalein	33.52	0.21
MOL002908	5,8,2′-Trihydroxy-7-methoxyflavone	37.01	0.27
MOL002909	5,7,2,5-Tetrahydroxy-8,6-dimethoxyflavone	33.82	0.45
MOL002910	Carthamidin	41.15	0.24
MOL002911	2,6,2′,4′-Tetrahydroxy-6′-methoxychaleone	69.04	0.22
MOL002913	Dihydrobaicalin_qt	40.04	0.21
MOL002914	Eriodyctiol (flavanone)	41.35	0.24
MOL002915	Salvigenin	49.07	0.33
MOL002917	5,2′,6′-Trihydroxy-7,8-dimethoxyflavone	45.05	0.33
MOL002925	5,7,2′,6′-Tetrahydroxyflavone	37.01	0.24
MOL002926	Dihydrooroxylin A	38.72	0.23
MOL002927	Skullcapflavone II	69.51	0.44
MOL002928	Oroxylin a	41.37	0.23
MOL002932	Panicolin	76.26	0.29
MOL002933	5,7,4′-Trihydroxy-8-methoxyflavone	36.56	0.27
MOL002934	Neobaicalein	104.34	0.44
MOL002937	Dihydrooroxylin	66.06	0.23
MOL000358	Beta-sitosterol	36.91	0.75
MOL000359	Sitosterol	36.91	0.75
MOL000525	Norwogonin	39.40	0.21
MOL000552	5,2′-Dihydroxy-6,7,8-trimethoxyflavone	31.71	0.35
MOL000073	Ent-Epicatechin	48.96	0.24
MOL000449	Stigmasterol	43.83	0.76
MOL001458	Coptisine	30.67	0.86
MOL001490	Bis[(2S)-2-ethylhexyl] benzene-1,2-dicarboxylate	43.59	0.35
MOL001506	Supraene	33.55	0.42
MOL002879	Diop	43.59	0.39
MOL002897	Epiberberine	43.09	0.78
MOL008206	Moslosooflavone	44.09	0.25
MOL010415	11,13-Eicosadienoic acid, methyl ester	39.28	0.23
MOL012245	5,7,4′-Trihydroxy-6-methoxyflavanone	36.63	0.27
MOL012246	5,7,4′-Trihydroxy-8-methoxyflavanone	74.24	0.26
MOL012266	Rivularin	37.94	0.37

**Table 13:** Common targets of botanical drugs and cancer pain diseases.

141 common target proteins						

ACHE	CD40LG	EGFR	HRH1	MAPK14	NR1I2	RAF1
ACTB	CES1	ERBB2	HSD3B2	MAPK8	NR3C1	RASA1
ADRA1A	CHEK2	ESR1	HSP90AA1	MDM2	NR3C2	RB1
ADRA2A	CHRM2	ESR2	HSPB1	MET	ODC1	RELA
ADRA2C	CHRM3	F3	HTR3A	MMP1	OPRD1	SCN5A
ADRB1	COMT	F7	ICAM1	MMP2	OPRM1	SELE
ADRB2	COX5A	FASLG	IFNG	MMP3	PCNA	SERPINE1
AKR1C1	COX6B1	FECH	IGF2	MMP9	PGR	SLC6A2
AKT1	CRP	FN1	IGFBP3	MPO	PIK3CG	SLC6A3
ALOX5	CXCL10	FOS	IKBKB	MT-CO1	PLAT	SLC6A4
AR	CXCL8	GABRA2	IL10	MTHFR	PLAU	SPP1
BAX	CYCS	GABRA3	IL1A	MTR	PON1	STAT1
BCL2	CYP19A1	GRIN1	IL1B	MYC	PPARA	THBD
BIRC5	CYP1A1	GRIN2A	IL2	NFE2L2	PPARG	TNF
CACNA2D1	CYP1A2	GRIN2B	IL4	NFKB1	PRKCA	TOP2A
CASP8	CYP27B1	GRIN2D	IL6	NFKBIA	PRSS1	TP53
CASP9	CYP2C9	GSTM1	IRF1	NOS2	PTGES	TYR
CAT	CYP3A4	GSTP1	JUN	NOS3	PTGS1	VCAM1
CAV1	DNMT1	HIF1A	KDR	NPPB	PTGS2	VDR
CCL2	EGF	HMOX1	MAPK1	NR0B1	PYGM	VEGFA
CCND1						

**Table 14:** Core target map of different parameters of botanical drugs cancer pain disease.

Degree value 30	Degree value 25	Degree value 20		Degree value 15		

TNF	TNF	TNF	CXCL8	NR3C1	MAPK1	MAPK14
MAPK1	IL6	AKT1	MAPK1	IL1B	NFKB1	IL4
JUN	MAPK1	RELA	EGFR	TNF	RELA	ESR1
	AKT1	JUN	MAPK14	IL6	EGFR	HSP90AA1
	RELA	VEGFA	ESR1	MAPK8	JUN	TP53
	JUN	TP53	HSP90AA1	CXCL8	VEGFA	
	HSP90AA1	IL6		AKT1	FOS	
	TP53					

## Data Availability

The datasets used and/or analyzed during the current study are available from the corresponding author on reasonable request.
